# The Deep Integration of China's Regional Ice-Snow Industry and Ecocultural Tourism under the Background of Beijing Winter Olympic Games: Taking Hunan as an Example

**DOI:** 10.1155/2022/6736709

**Published:** 2022-07-11

**Authors:** Wu Lingmin, Feng Haitao

**Affiliations:** ^1^Hunan Institute of Engineering, Xiangtan 411004, China; ^2^Hebei University of Science and Techology, Shijiazhuang 050018, China

## Abstract

Under the background of the promotion of the Olympic effect of the 2022 Beijing Winter Olympics and the in-depth implementation of the national ice and snow industry's strategy of “expanding from the south to the west and expanding from the east,” China's ice and snow industry has ushered in a new period of development. By applying literature and logical analysis, etc., with in-depth analysis of various subjective and objective supplies for the integration of China's ice-snow industry and ecocultural tourism in Hunan Province, it is considered to be driven by the bidding and preparation effect of Beijing Winter Olympic Games in 2022. The supply capacity of ice-snow industry venues, professional facilities, and public services are gradually strengthened, and the soft power of construction of the ice-snow industry needs to be coordinated and improved. The problem of safety is prominent and it is urgent to build a safety prevention and emergency management of ice-snow tourism.The integration of ice-snow sports and ecotourism industry has gradually became a prototype, but the integration point, line, and surface still need to be further strengthened and expanded. Accordingly, this paper puts forward a method to realize the transformation and upgrading of the commercial operation mode of the integration of ice-snow industry and ecological culture tourism, comprehensively to improve the ecological innovation ability of ice-snow tourism public service, to create multi-industry ice-snow industry cluster area, and to construct the basic framework system of risk prevention and control and management with multisubject participation and other relevant strategies.

## 1. Introduction

With the full implementation of the preparation and successful holding of the Beijing Winter Olympics, the effect of the Winter Olympics on promoting the regional ice-snow tourism industry industry is being fully released. Under the background of the new era of symbiosis, sharing and win-win tourism economic development, ice-snow tourism industry, as a new form of tourism development with ecological, economic, cultural, integrated, protective, and systematic attributes, is an important part of the most dynamic and potential sunrise industry, white industry, health industry, and people's livelihood industry in the world-recognized regional tourism [1]. In view of the obvious attribute characteristics of the wide range and strong driving force of the ice-snow tourism industry, this industry is becoming a booster to promote the high-quality development of global tourism [2].

The prominent green, low-carbon, safe, and balanced attributes of ec-tourism fit the harmonious coexistence of ice and snow industry development and society, human beings, and nature. The deep integration of ice and snow tourism and ecotourism is the historical necessity to realize the sustainable development of the ice and snow tourism industry [3]. However, the integration time of regional ice and snow industry and ecocultural tourism in China is relatively short and the integration products are highly qualified with the market. The integration mechanism and system are also in an urgent need of reform and improvement [4]. Based on this, standing on the concept of new development, this paper interprets the current situation and existing problems of the integration of regional ice and snow industry and ecological culture tourism in China with typical cases and puts forward the choice of an innovative path, which has certain practical significance and theoretical value for alleviating the various contradictions between the demand and supply of regional ice and snow production, promoting the transformation and upgrading of regional ice and snow industry, and promoting the in-depth implementation of the strategy of “south development, west expansion, and east development” of China's ice and snow industry.

## 2. Research Objects and Methods

### 2.1. Research Objects

Taking Daweishan Ski Resort, Dongshanfeng Ski Resort, Three Bear Ski Resort, Liuyang Ruixiang Ski Resort, and Changde Taohuayuan Ski Resort in Hunan Province as investigation objects, the integration of skiing industry and regional culture, architecture, commerce, and trade is the main investigation content. This paper conducts in-depth analysis from two aspects: the supply of ice and snow industry itself and its integration with related industries.

### 2.2. Research Methods

#### 2.2.1. Mathematical Statistics

The obtained data were processed with the commonly used statistical methods such as the average, standard deviation, and single sample-t test of Microsoft-Exeel2017 and SPSS20.1 in OFFICE2017.

#### 2.2.2. Questionnaire Survey Method

The methods are as follows: (1) Questionnaire design and testing. According to the relevant literature, combined with the practical needs of this study, this paper constructs the index system of ski industry supply capacity and integration with other industries in Hunan Province. Through two rounds of expert interviews and adjustments, the validity of the questionnaire is ensured to be greater than 80%. (2) Questionnaire survey and recovery. Using cluster sampling, five ski resorts currently operating in Hunan Province were selected as the survey objects and field research methods were adopted. Through paper questionnaires and face-to-face interviews with ski resort managers, the actual situation of each index in the supply of ice and snow tourism and its integration with other industries were collected. Five questionnaires were sent out with a recovery rate of 100%.

#### 2.2.3. Strategic Transplantation Method

With the combination of strategic transplantation and strategic innovation, this paper studies the realization path of deep integration of ice and snow sports industry with other industries.

## 3. Objective Basis of Promoting Integration of Regional Ice-Snow Industry and Ecological Culture Tourism in Beijing Winter Olympic Games

### 3.1. The Construction of Ice-Snow Industry Venues and the Supply Capacity of Ice-Snow Industry Supporting Facilities Gradually Increase

Influenced by natural geography and climatic conditions, the development of ice-snow industry sports for the masses in the south of the Yellow River in China is hindered by more realities [5]. The supply of ice-snow industry venues and facilities is the basis for the integration of ice-snow industry and ecological culture tourism. Regardless of the number and scale of ice-snow industry venues in southern China, there is a big gap with the north [6].With the radiation effect of the Winter Olympics and the demonstration effect of Ye Qiao-bo, Yang Yang, and other athletes on the contemporary social economy, culture has had a profound impact and the strategic needs of the development of China' government ice-snow industry sports; China's ice-snow industry sports southward expansion and eastward into the area venues supply capacity increased year by year. By the end of 2020 [7], there were 770 ski resorts in China. There were 28 new ski resorts in China, including 5 indoor ski resorts, with a total of 770, an increase of 3.77%. At present, there are 9 ski resorts in Hunan Province (including 2 outdoors) and 3 ski resorts under construction (Wu Gaishan Ski Resort, Chenzhou; Wang Yunshan Ski Resort, Shaoyang; Heng Fengshan Ski Resort, Hengyang). Ski resort's infrastructure and professional facilities are inadequate in Hunan Province, whether it is the length of the magic blanket, or ski press, the number of high-altitude cableway, and the national average, there are significant statistical differences (see Table 1).

As can be seen from Table 1, at present, the outdoor ski slopes in Hunan province are mainly set up with primary and intermediate trails, without professional trails. However, the limitation and lack of hardware conditions of magic carpets and high-speed cable cars cannot provide ice-snow industry tourists with better emotional experience of controlling the ice-snow industry. To some extent, it also limits the resource space for ice-snow industry tourists to change from tourism experience type to learning type and even vacation type. In a relatively competitive environment, lack of professional facilities will exacerbate the competitive disadvantage of ice-snow industry enterprises. At present, the outdoor ski resorts in Hunan Province are basically located in the countryside, lacking high-speed rail and air express transportation, and there are basically no tourist buses and direct public transportation in the ski resorts. This traffic barrier connecting the ice-snow tourism industry destinations and the tourist source areas undoubtedly limits the ice-snow industry tourist sources to specific target groups and cannot attract other ice-snow industry enthusiast groups in the region. Although some indoor ski resorts have a small part of the bus directly reached, such as Rui Xiang Ski Resort in Hunan Province, the ski resort also cooperates with the travel agency, launched the indoor ice-snow tourism industry line; there are also special tourist routes. However, most of the ski traffic inconvenience to a certain extent limits the development of ice and snow industry in Hunan Province. On the other hand, the outdoor ski resorts in Hunan Province operate in winter, and the summer ski resorts are in a state of waste, resulting in idle and waste of resources. The management of the European ice-snow industry has experienced a hundred years of development [9]. At present, the focus of ice-snow industry development in various ice-snow industry regions is not on the number and scale of snow fields, but on the upgrading of services and supporting facilities between snow fields and improving the customer experience of tourists to win tourists. Therefore, to promote the high-quality development of the integration of ice-snow industry and ecological and cultural tourism in the South Expansion, West Expansion, and East Expansion area of the ice-snow industry sports, it is necessary to rely on the natural ecological environment conditions of the ice-snow industry venues themselves to avoid the destruction of the ecological environment caused by the construction of large-scale ice-snow industry venues. With the supply efficiency of green, low carbon, and systematic circulation of ice-snow industry venues, the existing infrastructure and professional supporting facilities should be updated and upgraded in a timely manner to improve the maximum utilization rate of the ecological development of the existing venues, and to meet the new needs of the integration of ice-snow industry and ecological and cultural tourism by improving their own soft indicators.

### 3.2. The Public Service Construction of the Integration of the Ice-Snow Industry and Ecological Culture Tourism Has Been Gradually Improved and There Is Great Room for Improvement in Human Resource Construction

Table 2 shows the current status of public service construction of ice and snow industry and ecological and cultural tourism integration in Hunan Province at present. It can be seen from Table 2 that the public service of ski resorts is based on the survey of six ski resorts (two outdoors and four indoors) in Hunan Province, and 2/3 of the ski resorts have professional qualification coaches generally between 4 and 6, while the number of professional coaches in some indoor ski resorts (open for the whole year) reaches 10–15, which cannot meet the tourism demand in the peak season of the ice-snow tourism industry. In terms of training time, there is no professional continuing education for employees in indoor ski resorts in Hunan Province, and the training time of indoor ski resorts is relatively short. The training of skiers in Hunan Province has not yet formed a systematic framework and system. From the safety staffing point of view, Hunan Province ski resort safety personnel, there is a lack of professional doctors. In response to epidemic diseases and medical emergencies, public health supply is insufficient. From the perspective of volunteer service, there is no ice-snow industry volunteers in ski resorts in Hunan Province and there is no participation of social welfare forces. Since skiing requires high skill and safety, especially in the south, west, and east of China, it is the first time to contact the ice-snow industry. Skiers need a professional personnel to guide their postures and skills, and the serious shortage of personnel undoubtedly poses a hidden danger to the safety of ice-snow tourism industry [10]. Ice-snow tourism industry, as a form of tourism industry with high seasonal dependence, has the largest loss of professionals among all tourism modes. In this survey, it is found that in the outdoor ski resorts in Hunan, the loss rate of ice-snow industry personnel is as high as 75%. Therefore, to promote the high-quality development of ice-snow industry in Hunan Province, we must pay attention to the cultivation of human resources and innovate the public service system of ice-snow industry venues.

### 3.3. Integration of the Ice-Snow Tourism Industry and Other Industries

The ice-snow tourism industry is a new sports tourism industry with the characteristics of ice-snow resources and tourism industry produced by the cross-integration of ice-snow tourism and other industries [11]. The integration of ice and snow industry is the mutual connection between internal or external industries of ice and snow tourism, which permeates each other and forms a new industrial system [12]. Pan believed that the integration of tourism industry includes the formation process of a core industrial chain and extended industrial chain^6^. From the internal point of view of the ice and snow industry, as a type of tourism, the ice and snow tourism industry is inseparable from the six elements of tourism (food, housing, transportation, tourism, entertainment, and shopping). From the external point of view, the ice and snow industry is closely related to the service industry, agriculture, and manufacturing. In the integration of ice and snow industry and other industries, the construction of a core industrial chain and extension industrial chain of ice and snow industry are the main manifestations. In this complex system, the integration of ice and snow industry should first consider the integration of ice and snow sports with elements such as catering industry, hotels, shopping centers, and transportation. With the upgrading of ice and snow industry, the integration of ice and snow industry with manufacturing, construction and cultural industries will continue to strengthen. The development of ice and snow industry in southern China is relatively late. The first ski resort in Hunan Province opened in 2011, with a short operating time and low integration with other local industries. Far from meeting the needs of public tourism, Hunan indoor ice and snow tourism venues tourism product homogeneity degree is high, there is no characteristic ice and snow brand. From the perspective of tourists, the lack of characteristic ice and snow service supply will greatly reduce the value and attraction of regional ice and snow tourism industry [13]. From the survey data of vacation hotels, recreational facilities, and large-scale buildings around the ice and snow tourism scenic spots, it can be seen that the number is very small and the construction is loose. Compared with the large-scale and cluster development of ice and snow tourism industry in the core area of ice and snow tourism, the ice and snow tourism market is highly homogeneous and lacks high value-added and regionally influential characteristics of ice and snow tourism products. On the other hand, from the ice and snow tourism marketing culture, the number of ice and snow performance is small, low level, just as a means of marketing and did not form the internalization of the fixed culture; the way of financing is single and there is a big gap in the construction and maintenance funds of ice and snow tourist attractions. At present, the integration of ice and snow sports industry with culture, tourism, food culture, architectural culture, and performance industry is low. Especially in the extension industry, China is also at a low level. In terms of Chinese ice and snow equipment manufacturing industry, according to Chinese Ski Industry Development Report 2019, the output value of Chinese sports goods industry reached CNY 307.7 billion in 2016, with an increase of 11.65% over the same period. As an important part of the sports industry, the ice and snow sports industry has great development potential but low market share. At present, most of China's ski equipment depends on imports. In terms of skiwear, snowboards, and other products, imported brands occupy most of the total high-end market [14]. Therefore, the challenge of how to extend the types of ice and snow industry and realize the integrated development of ice and snow industry and other industries on the basis of highlighting the characteristics and highlights of the existing ice and snow industry development is an urgent problem for ice and snow enterprises, and also an objective requirement for the transformation and upgrading of China's ice and snow industry. In order to explore the new direction of the development of the “South Station West Expansion and Eastward” area of the ice and snow industry, it is necessary to cultivate the deep integration market of the ice and snow sports industry and other industries, create a new pattern of the deep integration of the ice and snow sports industry and other industries, promote the innovative development of the deep integration of the ice and snow sports industry and other industries, and stimulate the new kinetic energy of the deep integration of the ice and snow sports industry and other industries.

### 3.4. The Ecological Security Construction of the Ice-Snow Tourism Industry in Hunan Province Ushers in a New Period of Development

With the bid to host the 2022 Beijing Winter Olympic—Zhangjiakou Winter Olympic radiation effect, China' ice-snow tourism industry ushered in the golden decade of rapid development. However, the sudden public security crisis during 2019–2021 had a negative and profound impact on the tourism industry [15]. The ice-snow tourism industry has stopped in an all-round way and China's ice-snow industry has suffered a cliff-like hit. According to the report on the market consumption survey and development strategy of China' tourist attractions industry from 2020 to 2026 issued by the Intelligent Research Consultation in April 2020, it shows that the loss of tourism in 2020 is more than 500 billion, of which the ice-snow industry is a serious disaster area. All outdoor and indoor ski resorts in Hunan Province were closed in 2019 and 2020, and the outdoor ski resort missed almost the whole tourist season. Public safety has become a key factor affecting the normal operation of tourism purposes in China. At present, the Chinese government, in cooperation with medical institutions around the world, has constructed a risk-level-based and regional progressive prevention and control strategy of China + neighboring countries + the world, which provides a new peripheral barrier for the orderly flow of personnel in the tourism industry [16]. China has established a prevention and control alliance involving the government, tourism communities, health departments, and other functional departments, and achieved top-down command, bottom-up feedback channels, and joint defense and control of different departments. Based on information, tourism communities integrate community resources to achieve fine management, scientifically plan the tourism capacity and tourism reception of scenic spots, effectively implement the identification, diagnosis, tracking, screening, isolation, and transfer of infectious diseases, and gradually move towards community intelligent prevention and control mode. However, China has not yet introduced a social-oriented evaluation and early warning mechanism for ecological security of tourism destinations with relevant standards and supervision capabilities; there is a lack of ecological security of ice-snow tourism industry venues, medical security of ice-snow tourism industry venues, ecological security of human management of ice-snow tourism industry, ecological security of tourism behavior and natural load, and the administrative intervention is also slightly thin. Therefore, in the post-epidemic era, building a deep integration prevention and control system of ice-snow industry and ecological tourism faces multiple challenges.

## 4. Discussion and Analysis

### 4.1. Accelerate the Transformation and Upgrading of Business Operation Mode of Integration of the Ice-Snow Industry and Ecocultural Tourism

Ice‐snow industry is an information intensive industry type. The complexity of the ice-snow tourism industry market and the details of tourism products containing information components affect and determine the share of the ice-snow industry [17]. The uniqueness of ice-snow tourism industry products and the formation of information and value chains are usually a mixture of products and services provided by different ice-snow tourism industry and related companies [18, 19]. After nearly 20 years of development, China has become the world's largest primary market of ice-snow industry. However, China's ice-snow tourism industry product market has a high degree of homogenization, and the uniqueness of ice-snow tourism industry product information is low. The tourism products provided by ice-snow industry industrial parks or ice-snow industry towns are basically dominated by winter operation. The supply of ice-snow industry products in China cannot meet the demand of four-season tourism, and the single-season operation mode also causes a great waste of resources. Based on this, it is necessary to accelerate the transformation and upgrading of the business operation mode of ice-snow tourism industry from one season type to four-season type industry (see Figure 1). Building a multi-industry ice-snow industry ecological industry cluster area is not only the objective requirement to solve the bottleneck of the development of ice-snow tourism industry industry in China but also the inherent demand for the sustainable development of green economy in regional ice-snow tourism industry ice-snow industry. The skiing industry requires a large investment and a relatively long capital recovery, especially in developing China's ice and snow industry planning “from the North to the South of China.” Due to the short snow season and the lack of tourism projects around the ski resort in spring, summer, and autumn, it is inevitable to have a huge waste of infrastructure and professional facilities around the ski resort. Especially in the years from 2020 to 2022, when COVID-19 is raging, it causes a sharp drop in the revenue of snow and ice tourism. Therefore, the winter operation mode of ski resorts in this region has disadvantages, and it is urgent to expand and innovate ice and snow tourism products. Second, from the perspective of business operation law, four-season tourism is more likely to attract investment and financing motivation and investment in industries such as food, real estate, hotels, and ecology and realize the deep integration of ice-snow industry and ecological tourism. In foreign countries, many super-large ice-snow industry resorts have already completed the transition from one-season tourism to four-season tourism. In particular, many super-large snow resorts in Europe have opened up new business projects through various channels and broke through the business constraints. Taking the Norwegian Winter Olympics hosting Hashan of Norway as an example [20], the local government transformed the Hashan ski resort after the Olympics. The Hashan Resort has perfect ice-snow industry service facilities, and there are ski shops at the entrance to provide all the equipment needed for ice-snow industry tourists. Norwegian resorts have good snow trails, mountain rope ways, and holiday villas. Tourists can return directly to the mountain resorts through high-speed rope ways. Resort villas provide Norway with local characteristics of food and all modern equipment, local tourism enterprises use winter tourism, other seasons to carry out bicycles, to achieve the four seasons of ice-snow tourism industry business and formed a complete, highly developed, perfect industrial chain. The development of ice-snow tourism industry in Hunan Province should rely on its own resources to create a four-season tourism business model. Spring operation: According to the characteristics of regional climate in spring, tourism is integrated into the protection of red, ancient books, and heritage, and the deep integration of indoor ice-snow tourism industry, outdoor leisure and red tourism, heritage tourism, and research tourism is realized. Leisure tourism in ice-snow tourism industry destinations is strengthened, and tourism commerce, tourism manufacturing, tourism real estate, and other industries are cultivated. Summer operation: Through the deep integration with modern sports culture and folk sports culture, taking the construction of cultural and tourism projects as the starting point, we gradually realize the deep integration of leisure sports in ice-snow tourism industry destinations with characteristics of Hunan folk culture and modern sports culture, expand the new format of tourism, create rock climbing, bicycle, drifting, folk tourism projects, and cultivate tourism commerce industry, tourism manufacturing industry, and other types. Autumn operation: Relying on regional heritage culture, modern, and folk culture, actively carrying out cross-border cooperation with sports tourism, competition, business, and other industries, and creating the characteristics of marathon and bicycle lamp outdoors. Winter operation  :  excavate modern winter Olympic culture, competition culture, folk culture, science and technology elements, increase the deep integration of ice and snow sports and regional culture, create ice and snow + manufacturing industry, ice and snow + performance industry, ice and snow + high level events, ice and snow + folk culture, ice and snow leisure tourism, and other ice and snow products, cultivate ice and snow industry with regional architectural culture characteristics, ice and snow commerce with regional characteristics, ice and snow events represented by large events, etc., to promote the deep integration and innovation development of ice and snow industry and other industries.

### 4.2. Build a Comprehensive, Three-Dimensional Integrated Security System of the Ice-Snow Industry and Ecocultural Industry

Ice-snow tourism industry is a complex system with specific structure, function, and goal. It is a complex system involving social, economic, and environmental factors. It has its own spatial structure, time structure, and space-time structure. The exchange and normal operation of energy, material, and information with the outside world can be realized only by maintaining stable interrelation and orderly interaction among the elements of the system [21]. Ice-snow industry and ecocultural tourism is a complex and comprehensive business operation, facing challenges from natural environment, society, human management, partnership, and other aspects. The optimization of ice-snow industry and related industries is the process of system components and system management to achieve the best state, in order to maximize the function of the system and achieve the best results. Under the background of national ecological civilization construction, tourism power and multiwheel drive development of Beijing Winter Olympic Games, the integration and ecological development of ice-snow tourism industry and related industries is historically inevitable. Regions have created different natural, cultural, and historical conditions and also bred characteristic tourism civilization. Regional tourism industry in turn has effected regional spatial, economic, and environmental changes. As an element of reshaping regional brand and image space tourism civilization, these tangible and intangible cultural heritages have a considerable development potential in the development of strategic tourism products and also reflect the characteristics and regional advantages of space tourism. Evolutionary psychology believes that as individuals are attached to a tourist destination, tourists will have a stronger desire to protect the region [22]. Managers of tourist destinations can make use of the social psychological interaction of tourists to assist in the sustainable management of tourist destinations.

Hunan province is the birthplace of Huxiang culture. After thousands of years of historical and cultural breeding and practice, Hunan Province has formed unique sports, food, architecture, drama, folklore, manufacturing, and other characteristics of culture. It can be said that these regional tourism superstructures, as well as the creation of tourism products on the basis of multilevel and more complex tourism attraction, are more likely to realize the sustainable development of the tourism industry. To achieve the integration of regional ice-snow industry and ecological culture in Hunan Province, it is necessary to reflect the regional spatial characteristics and advantages, organically combine Hunan civilization with ice-snow industry and ecological civilization, realize ecological guidance, continuously coordinate the relationship between economic benefits and environment, and provide effective supply of ecological ice-snow tourism industry experience and related tourism ecological services for sports tourists. From the perspective of time dimension, the integration of ice-snow industry and ecocultural tourism should also undergo a dynamic periodic process of germination, development, consolidation, stagnation, decline, and revival. All aspects and stages of industrial integration are intertwined and continuous. At different stages, the integration of ice-snow industry and ecological culture tourism shows different risk conditions. The challenge of how to solve the problems in the integration of the two needs to rely on the extensive and reliable information data of the fusion destination. On the other hand, time dimension can also be understood as a social structure and operational structure. Foreign research shows that in the process of deep integration of the two, it is increasingly dependent on the coordinated participation of technology, organization, and other changes, especially marketing activities and management. Tourism, as one of the largest industries in the world, has significant social, environmental, economic, and political implications. Its own spatial and temporal structure characteristics show that the impact of tourism development is far more complex than what decision makers usually say. The impact of tourism not only occurs in destinations but also occurs at all stages of tourists' travel. The integration of ice-snow industry and ecocultural tourism is affected and restricted by broader social and environmental changes. It is also destined to the continuous adaptation and adjustment process of ice-snow tourism industry and related industries, select a reasonable integration model, and enhance the operational potential of local tourism planning and management departments.

Objectively speaking, it is complex to accelerate the integration of ice-snow tourism industry and ecocultural tourism, which not only needs to be promoted from the aspects of government policy support, cultural derivation of ice-snow tourism industry, and industrial technological progress but also needs to be driven by innovation of strategic opportunities of Beijing Winter Olympics. First of all, the Beijing Winter Olympics can not only provide a huge market space for China to promote the upgrading of the ice-snow tourism industry industry itself but also provide important support from the regional ice-snow industry venues and the landing of ice-snow industry. projects. It can form a strong impetus for the upgrading of regional ice-snow tourism industry industry to promote the sustainable development of regional ecological economy from the transformation of government management functions and the consumption concept of public ice-snow tourism industry. Second, as a sunrise industry with high correlation, strong driving force, vigorous vitality, and great growth potential, ice-snow tourism industry will also become an important foundation and driving force to promote regional ecological and economic development under the incentive of Beijing Winter Olympics. At the beginning or earlier stage of industrial development, various factors should be comprehensively considered, and the protection of the ecological environment should be implemented in the whole tourism industry and its subsidiary industries, as well as the continuous adjustment and optimization system construction, that is, the ecological function should be implemented in the whole process of tourism industry and related industries, and the ice-snow industry and related related industries should be specifically implemented. Its management and operation should highlight the ecological development direction and implementation path from the aspects of enterprise planning, product marketing, human resources management, and so on. In the integrated development of ice-snow industry and ecotourism, the government should cooperate and interact with tourism enterprises and nonprofit organizations in advance. From the formulation of ecological policies, implementation in supervision, reward, and punishment, the government should innovate the theory and method of tourism public service to explore and innovate the way, service system, service organization, service concept, and service function of tourism service and establish a new performance evaluation system to make the government's public service work measurable. The government should actively build a communication bridge between the tourism industry and related industries and the people, mobilize the national social media force, and carry out multidimensional low-carbon, environmental protection, safety, and balanced ecological national education.

### 4.3. Construction and Improvement of a New Public Safety Service System for the Integration of the Ice-Snow Industry and Ecocultural Tourism

The public service of ice-snow tourism industry scenic spot is an important supply factor of ice-snow tourism industry destination, and it is the core index parameter in the construction of modern ice-snow tourism industry brand. It reflects the soft power level of modern ice-snow tourism industry brand and the core competitiveness of tourism products. In a modern society full of competition and rapid growth, tourism itself and tourism demand are changing rapidly. New technologies, more experienced consumers, global economic restructuring,, and damage to the ecological environment pose some challenges to the industry. Compared with the super regions of ice-snow industry in Europe and America, the supply of China's ice-snow tourism industry is more manifested in the limitations and deficiencies of tourism service level and ability. From the domestic point of view, in addition to the gap between the scale of ice-snow tourism industry, tourist reception, and other quantitative indicators, the reception capacity and service level of ice-snow tourism industry scenic spots in China are also different from those in the north. Especially with the continuous deepening of the integration of ice-snow industry. and ecological culture tourism, the quality and efficiency of public services in ice-snow industry and related industries are higher. From the perspective of tourism public security services, the international spread of new pneumonia from the end of 2019 to 2020 has a significant impact on the world tourism economy. The expectation for the ecological security of tourism and related industries in society can be said to exceed all periods of history. From the perspective of ice-snow tourism industry itself, at present, the participation mode of ice-snow tourism industry in China is also changing from the ice-snow tourism industry of the travel agency team to the self-help tourism of the destination. The personalized, popular, scattered, and normalized trend of ice-snow tourism industry activities is becoming increasingly obvious. This kind of change causes the passenger to the ice-snow industry tourist scenic spot security, the ice-snow industry tourist scenic spot information release and provides the ice-snow industry tourist scenic spot traffic guidance service demand to be stronger. At the same time, with the continuous improvement of people's participation in southern ice-snow tourism industry activities, tourists' awareness of rights protection is increasing. Visitors for snow and ice tourism scenic safety complaints, snow and ice tourism information and self-driving tour services, snow and ice tourism scenic information, and other public service platform requirements are also increasing. Based on the above changes in security, technology, and demand, it is urgent for the current ice-snow industry enterprises to upgrade public tourism services.

Under the background of globalization, the supply of public services for the integration of ice-snow industry and ecological culture tourism in China has undergone profound changes, and the traditional tourism public service practice has also become more humanized and fragmented. The construction of public services for the integration of ice-snow industry and ecological culture tourism is a huge, complex, and dynamic system. Its supply includes various forms of government, market, and social organization, which requires the establishment of a variety of cooperative mechanisms for governance subjects. This process is usually manifested as a dynamic system formulation and implementation process. With the deepening of the integration of China's ice-snow industry and ecological culture, the public service of China's ice-snow tourism industry destination has undergone unprecedented changes. China's ice-snow industry and related industries are more dependent on technology supply, which is not only reflected in the efficiency and scope of professional services, medical security, health, and safety guarantee network supply but also reflected in the connectivity of tourism traffic, in advance payment, marketing, catering, hotels, and other aspects. The ice-snow industry and related industries in the new era of public service requirements also need to re-bound government, market, and social relations. The state's public service function of tourism destinations has gradually transited and transferred to the market-oriented supply mode, and the state supply has begun to shift from dominance to regulation. The government intervenes in the level and quality of public services in ice-snow tourism industry areas through market access, service quality, and interval regulation. In the process of forming this goal, the government provides subsidies in the form of state payment for parts that are difficult to bear by enterprises, so as to ensure that public services meet the increasing public demand for tourism destinations. By innovating the regulatory mechanism of tourism public services and other legal construction, the state optimizes the efficiency of tourism administrative services and provides strong policy support and effective supervision for the integrated development of enterprises. In terms of public services of China's ice-snow industry enterprises, according to the higher requirements of the technical specifications of the market-oriented management of public services, it is necessary to improve the construction of the standardization system of tourism public services in a timely manner, optimize the tourism public service environment, and use scientific and technological means to build a network service platform, so as to provide data support for the integration of ice-snow industry. and ecological and cultural tourism, so that society and consumers can use the network service platform to rating and comment on the tourism process, so as to better improve their services and provide a convenient, safe, fast, and green service for ice-snow industry tourists.

### 4.4. Build the Risk Prevention and Control Security System of the Ice-Snow Industry and Ecological Culture Tourism Integration

The prevention and control of ice and snow tourism is an important guarantee for the sound operation of ice and snow tourism. Based on Feng's ice and snow tourism prevention and control model [23], combined with Zhang and Qiyan's implicit integration period, explicit integration period and promotion integration period' integration staging theory of tourism integration [24], this study constructs the basic framework system of risk prevention and control of ice and snow sports and ecological tourism integration.

It shows the key factors of tourism prevention and control in different periods of the integration of ice and snow sports and ecological and cultural tourism. From Figure 2, we know the prevention and control of internal and external risks in the integration process must involve the joint participation of multiple departments in China. From the perspective of the subordinate relationship of the ice-snow industry is directly managed by the local tourism bureau, and its ice-snow industry planning is affected by the overall layout of the Ministry of Culture and Tourism. The investment and tax concessions for the integration of the ice-snow industry with other industries are subject to the direct jurisdiction of the Ministry of Finance and the State Administration of Taxation. In addition to the national finance, the funds and support for the integration of ice-snow industry and related industries are also derived from the investment and financing of social forces. The risk prevention and control of ice-snow industry is also subject to national audit and social supervision. Ice-snow industry enterprises are the direct implementer of risk management and control of industrial integration. They are directly subject to the management of board functional departments and regulatory authorities and are responsible for the daily affairs' management of the integration of ice-snow industry and ecological and cultural tourism. From the ice-snow industry, management structure is not difficult to see; risk management is a complex system engineering, capital, management, science, and technology have an immeasurable impact on the tourism industry. Therefore, the construction of a basic framework for risk prevention, control, and management involving the state, society, and enterprises is also an important method and means to realize the integration of ice-snow industry with other industries. On the risk prevention and control in the early stage of integration, it is usually based on the comprehensive evaluation of the state to realize the overall planning and infrastructure construction layout of the integration of the ice-snow industry and related industries and rely on policy and financial advantages to reasonably plan and effectively avoid the potential risks of the integration of the two. The relevant departments in charge of the integration of ice-snow industry and related industries mainly analyze and sort out the feasibility analysis, integration objectives, and subjective and objective basis of integration, providing reference data for the overall planning of national integration. It can be said that in the early stage, the state plays a leading role in the prevention and control of the integration risk of ice-snow industry and eco-cultural tourism. Trade associations and other social forces carry out effective and close supervision and implementation of the integration of the two in accordance with the relevant national policies and overall planning. With the deepening of the integration of ice-snow industry and ecological culture tourism and the initial appearance of industrial integration, the role of internal management of ice-snow industry enterprises in the integration of the two is becoming more and more obvious. The integration of ice-snow industry and eco-cultural tourism relies more on the internal control of tourism enterprises to obtain more external information, while the internal control evaluates the integrated risk of the integration of the two from the control environment, risk assessment, control activities, information and communication, and monitoring, which in turn improves the effectiveness of the overall internal control of the integration of the two.

With the deepening of integration, the integration system and policy system of ice-snow industry and ecological and cultural tourism are further improved. The capital operation of ice-snow industry enterprises is more rational and standardized, and the role and status of science and technology are becoming more and more prominent. The integration of ice-snow industry and high-tech leads to a large number of new formats. The state gradually gives way to enterprise risk management, and the integration work is more completed through enterprises. From the development of the European ice-snow industry enterprises, it can be seen that in the late stage of the integration of ice-snow industry and local culture, ice-snow industry is more closely intertwined with culture, architecture, food, catering, and other elements. Industrial integration makes the independent industrial value chain partially or completely integrated, and new formats become a new driving force for regional economic development. Big data and artificial intelligence are more closely combined with these industries. Enterprises rely more on market rules, and risk early warning mechanism is more perfect and reliable.

From the current development trend of ice-snow industry. in Europe and the United States, the integration of ice-snow industry and ecological culture tourism will be more “human needs.” The risk of ice-snow tourism industry mainly focuses on service safety risk, ecological risk, and scientific and technological safety. The risk prevention and control of ice-snow industry enterprises pay more attention to the operational process, and the prevention and control is more institutionalized and operable. The ice-snow industry enterprises can more accurately analyze the current situation of organizations, environment, goals, tools, measures, and other factors and optimize the construction of early warning, supervision, evaluation, and control mechanisms. As the supervisor, the state uses policy advantages to further strengthen market supervision and enterprise operation supervision, so as to effectively avoid the existing and potential risks from the market and enterprises and form a solid defense barrier. However, the prevalence of new coronavirus pneumonia has brought an unprecedented impact on China and the world's ice-snow industry and has brought great challenges to the prevention and control of China and the world's ice-snow industry sports industry. Although the state and society have initiated emergency mechanisms and established a risk-based prevention and control strategy based on risk levels and regional gradual increase, top-down command, bottom-up feedback channels, and joint prevention and control of different departments in China + neighboring countries + the world, but unpredictable risks still exist. Therefore, in this sense, the construction of risk prevention and control system is still a long way to go.

## 5. Conclusion

To realize the great-leap-forward development of China's ice-snow industry, it is necessary to reform and adjust the following aspects: Firstly, on the basis of accelerating the construction of the dynamic mechanism of expansion of the south, west, and east of the construction of the ice-snow industry venues, improving the supervision and management subject, investment subject and the periodic effect of the construction of the regional ice-snow industry venues, the government's policy of promoting the construction of the ice-snow industry venues, market demand, construction funds, investment and financing methods, accelerating the self-upgrading of the regional ice-snow industry in the process of marketization, commercialization and informatization, and optimizing the industrial structure of the ice-snow industry. In order to improve the supply quality and efficiency of ice and snow industry, it is necessary to comprehensively improve the professional equipment and human resource allocation of ice and snow industry in the region; correctly handle ice and snow tourism product innovation and business model innovation. Increase the supply of public service products in ice and snow tourism attractions, in order to promote the development of China' s ice and snow industry in the south, west and east.. Second, it is necessary to resolve the shortage of funds for promoting the development of ice-snow industry's “expanding from the south to the west and expanding from the east” by the Beijing Winter Olympics, and to use a variety of models to promote the multicenter spatial integration of ice-snow industry, so as to realize the new situation formed by the Beijing Winter Olympics in promoting the development of ice-snow industry and promote the sustainable development of ice-snow industry expanding from the south to the west and expanding from the east.

## Figures and Tables

**Figure 1:** Ice and snow industry and ecocultural tourism integration framework.

**Figure 2:** Basic framework for integrated prevention and control of ice and snow sports and ecotourism.

**Table 1:** A list of the skiing infrastructure and professional supporting facilities of some ski resorts in Hunan province.

Name	Type	Magic carpet	Snow machine	Snow compactor	High-speed cable car	Snow road	Snow gear (set)	Communication	Transportation (near)
TaiWai Shan Ski Resort	Outdoors	500–600	16	1	No	Junior/senior	1000–1500	WIFI	County highway
Tung Shan Fung Ski Resort	Outdoors	500–600	12	1	No	Junior	1000–1500	WIFI	County highway
Three Bears Ski Resort	Indoors	300–400	1	1	No	Junior	1000–1500	WIFI	AIR/NATIONAL road/high speed rail
Shui Cheung Ski Resort	Indoors	300–400	2	1	No	Junior	1500–2000	WIFI	County highway
Fa Yuen Ski Resort		<300	1	1	No	Junior	500–1000	WIFI	County highway
The nation	In/outdoor	764/0.189	8	0.63	1.32	—	—		
		*P* < 0.05	*P* < 0.05	*P* < 0.05	*P* < 0.001				

Data as of December 2020—indicating no relevant statistics. The data of “ice and snow venues and supporting facilities construction” in the table are from the blue paper of the ice and snow industry edited by Beijing Carbin Institute of Ice and Snow Industry: China Ski Industry Development Report 2019–2021 [8].

**Table 2:** A list of staffing conditions of some ski resorts and other soft power in Hunan Province.

Name	Certificate Coach()	Management personnel	Snow field technology management professional	Professional training time (D)	Security personnel	Ambulance personnel	Volunteer	Emergency medical care	Drill security
TaiWai Shan Ski Resort	6	Lack	Lack	0	5	1	No	No	No
Tung Shan Fung Ski Resort	5	Lack	Lack	0	4	1	No	No	No
Three Bears Ski Resort	12	Lack	Lack	10	8	1	No	No	No
Shui Cheung Ski Resort	11	Lack	Lack	15	4	0	No	No	No
Fa Yuen Ski resort	4	Lack	Lack	10	3	0	No	No	No
Nation	—	—	—	—	8	0.63			—

Note: Indicates no data available until december 2021. The data come from the survey of the project group “Research on the Deep Integration of Regional Ice and Snow Sports and Ecocultural Tourism in China under the Background of Beijing Winter Olympics. “‐” means Lack of relevant data in authoritative literature.

**Table 3:** Basic information of ice-snow tourism operation in Hunan province.

Name	Project setting	Recreation place resort	Resort Hotel <5 KM	Products market <5 KM	Ice-snow publicity and promotion
TaiWai Shan Ski Resort	Skiing/entertainment projects	2	No	No	Bus poster publicity, national highway or expressway sign publicity, television, or Internet publicity.
Tung Shan Fung Ski Resort	Skiing/entertainment projects	0	No	No	Bus poster publicity, national highway or expressway sign publicity, television, or Internet publicity.
Shui Cheung Ski Resort	Skiing/entertainment projects	1	No	No	Bus poster publicity, national highway or expressway sign publicity, television, or Internet publicity.
Fa Yuen Ski Resort	Skiing	0	No	No	Posters or TV network publicity.

Note: Indicates no data available until december 2021. The data come from the survey of the project group “Research on the Deep Integration of Regional Ice and Snow Sports and Ecocultural Tourism in China under the Background of Beijing Winter Olympics.

## Data Availability

All the data contained in this study can be obtained by contacting the corresponding author. Readers can also inquire part of the original data and the results of data processing in this paper.
